The article "Analysis of News Dissemination Path and Impact of Big Data Technology in Public Health Emergencies" was retracted in 2023. Reasons: signs of a paper mill; suspected computer-generated content; unreliable results or conclusions; concerns about the data.

# Analysis of News Dissemination Path and Impact of Big Data Technology in Public Health Emergencies

**DOI:** 10.1155/2022/4436232

**Published:** 2022-08-30

**Authors:** Zhian Zhang, Jiayi Tang

**Affiliations:** ^1^School of Journalism, Fudan University, Shanghai 200433, China; ^2^Institute of Guangdong, HongKong and Macao Development Studies, Sun Yat-Sen University, Guangzhou 510275, China

## Abstract

Throughout the past public health early warning work, there is still a lack of early warning. Therefore, starting from the reform of the public health early warning mechanism, this paper sorts out the design and development of our country's public health early warning mechanism and its legal framework and further analyzes the unresolved problems that exist in early warning work. At this stage, our country's public health departments have put forward targeted suggestions for improving the early warning mechanism for emergencies and stabilizing public order. In this context, the following data are obtained: (1) The timeliness under the big data model is 73.81%, the prudence is 84.25%, the sustainability is 96.28%; the timeliness under the data mining model is 61.98%, prudence is 77.58%, sustainability is 83.24%; and the timeliness of the intelligent computing model is 53.44%, prudence is 65.58%, and sustainability is 96.28%. (2) During public health emergencies, the path of news dissemination includes 54 people for radio and television communication, accounting for 13%; 98 people for digital communication, accounting for 24%; 73 people for digital TV communication, accounting for 19%; the number of public relations companies was 63 people, accounting for 16%; the number of people who reprinted and spread was 52 people, accounting for 12%; the number of people who searched and spread was 73 people, accounting for 19%; the number of people who spread mobile phone messages was 32 people, accounting for 9%. At this stage, according to the characteristics of public health emergencies, the problems existing in the early warning work are analyzed, and specific suggestions for improving the early warning mechanism of public health emergencies in our country are put forward to stabilize the “public order.” Research in this area is ongoing.

## 1. Introduction

As a hot technical field, big data technology has received extensive attention and research, emphasizing the concept and nature of big data, development at home and abroad, as well as data collection and perception, storage and processing, data visualization and data analysis. Articles provide general information. Security and privacy practices, key technologies, and innovative technologies, identify the latest research directions of these technologies, summarize the technical and policy challenges of big data technologies, and review the application of their technologies to educational research and design applications [1]. Our country is currently focusing on the research on smart grid big data technology which has achieved many research results that mark the development of our country's power industry. So, once you understand the meaning of big data in smart grid, you will understand the concept of big data in smart grid, understand the key technologies and development trends of smart grid big data, put forward your own ideas and suggestions, and promote the correct application of smart grid big data [2]. The generation of big data brings new challenges to massive computing technology. In order to have a more comprehensive and in-depth understanding of the meaning of big data, this paper will examine the conceptual characteristics of big data, the overall processing process, and key technologies. The creation of this article is based on a brief description of the basic concepts of big data, a summary of the overall process of big data processing, and an introduction to the basic process and organizational structure of key technologies [3]. Big data is coming to us, and we are rapidly entering the Big Data Era. Big data requires freedom, transparency, and information sharing. Our time is also known as “shared time,” but we are also constantly under the control of a “third eye,” and with it comes intimacy. In the age of big data, mystical concerns about conservation raise questions of freedom and human responsibility, posing new challenges to traditional ethics [4]. The rapid development of big data technology provides operators with fast and massive computing solutions for traditional services (such as network design and optimization), and lays a solid foundation for operators to develop new services (such as credit scoring, personalized recommendation, and Internet services). This has important implications for the development of the industry. Research-related big data technologies provide background design best practices and key challenges for operators to apply big data technologies in the enterprise [5]. Rapid detection of public health events and rapid and effective reduction of morbidity and mortality have always been the work of public health focus. Loss or no financial loss, the current requirements become clear and necessary. Counting every second is required to respond to public health emergencies [6]. Public health emergencies have caused severe psychological stress and emotional problems for many people. In emergencies, psychosocial factors become increasingly important in guiding the investigation and emergency management process. Manifestations of emotional problems in emergencies include hypochondria, panic, anxiety, depression, and obsessions. Unexpected events provide ample opportunities to explore emotional issues [7]. The use of early warning to prevent and minimize emergencies such as natural disasters, accidents, and welfare events has a long history, but early warning of public health emergencies has not yet been carried out. Emergency regulations will monitor and give early warning to the business requirements of the content of the public health emergency plan [8]. A health emergency is a public emergency that causes or may cause serious harm to public health. These include, in particular, serious phenomena such as infectious disease pandemics, unexplained diseases, and major food and industrial poisonings. They affect public health (such as major environmental pollution, radioactive pollution, and major animal diseases), maintain public order and stability [9], learn more about developing public health emergency mechanisms, establish an effective management system for public health emergencies, develop a comprehensive online direct reporting system, strengthen the construction of grass-roots disease prevention and control systems, and establish a series of sensitive early warning mechanisms and reagents. They also strengthen on-the-job training and continuously improve the ability to respond to public health emergencies [10]. Understanding the characteristics of the online dissemination of alert messages is critical to managing alert situations and facilitating the dissemination of critical information, we will create a systematic and comprehensive analysis system combined with existing knowledge, to explore the unique evolution, dissemination, and common patterns of emergency knowledge dynamic [11]. Currently, the rapid development of online media and the continuous integration of traditional media has brought changes to the news dissemination mechanism. Although the communication efficiency has been greatly improved, there are still many problems. In particular, the dissemination of hot and negative news often brings controversy and negative impacts. This paper analyzes the current hotspot negative news dissemination mechanism, and proposes intervention paths, in order to provide a certain reference for monitoring the dissemination of negative news. It firmly grasps the positive direction of news dissemination [12] and describes a multi-channel dissemination system for online news articles on the Internet. This paper proposes the “value” of online news relative to the topic-time relationship, and a method for judging the topic expansion of the list of subsequent articles. Furthermore, we describe a method for reconstructing and presenting lists of time-series documents with high newsworthiness. Finally, a prototype system based on this method is described [13]. Globalization has had a profound impact on the news communication and news communication education in our country. In order to meet the requirements of the new era, our country's journalism and communication education needs innovation. This paper analyzes the influence of globalization on China's news dissemination and its influence on the cultivation of news talents. Some countermeasures for innovation in journalism and communication education in our country are analyzed from the aspects of changing educational concepts, adjusting curriculum settings, strengthening students' quality education, and strengthening the construction of teaching staff, providing a reference for the innovation of journalism and communication education [11]. China's modern information and communication enterprises are information and communication enterprises with Chinese characteristics. Politically, it is a part of the socialist cause led by the Communist Party of China; ideologically, it is derived from Marxist journalism; and economically, it is a commercial operation based on market operation to achieve hierarchical management and legalization [14].

The article "Analysis of News Dissemination Path and Impact of Big Data Technology in Public Health Emergencies" was retracted in 2023. Reasons: signs of a paper mill; suspected computer-generated content; unreliable results or conclusions; concerns about the data.

## 2. Public Health Emergencies

### 2.1. Overview of Major Public Emergencies and Their Handling

It can be seen from the data that our country's netizens are large in scale, spend a long time online, and have a high usage rate of new media such as short videos. The Internet has been deeply integrated into the public's life and work, affecting all aspects of public life. Our country has entered the Internet era. In recent years, public emergencies have occurred frequently. With the development of self-media, many public emergencies have been spread very quickly on the Internet, and they are very easy to ferment. Due to improper handling, many public emergencies have been used by some people with ulterior motives and become tools to intensify negative emotions, thus triggering online public opinion and even evolving into new public incidents, causing secondary harm. From the public reports in recent years, the author has sorted out the major public emergencies that occurred and their handling process, the network public opinion they caused, the consequences of the incident, and the results of accountability. Many incidents have learned a lot. Judging from the causes of major public emergencies in the past 20 years, the process of handling them, and the Internet public opinion caused, public health incidents, safety production incidents, social security incidents, natural disasters, etc. These incidents are easily handled improperly, leading to the spread of Internet rumors and public opinions.interact with each Although rumors have been refuted, information has been released, and illegal criminals have been cracked down, the cracks between the government and the public have to be closed through many efforts, and may even cause irreversible losses. Public emergencies are very likely to cause casualties and property losses, with great impact and harm. The “National Emergency Response Plan” defines general emergencies as: emergencies that cause heavy casualties, property losses, environmental damage, and serious social damage, and pose a threat to public safety. Public emergencies are mainly divided into four categories: natural disasters, accidents, public health events, and welfare events. Public emergencies are easily spread on the Internet, and their influence has gradually attracted people's attention. For a long time, all sectors of society have paid close attention to network security, strongly calling for the strengthening of cyberspace governance in accordance with the law, and calling for the introduction of laws related to network security. On June 1, 2017, our country's first cybersecurity law came into effect, clearly requiring that in the event of a cybersecurity breach, a cybersecurity emergency plan should be formulated immediately, an incident should be investigated and assessed, and network operators should take action to deal with potential security risks, prevent damage, and keep the public informed. At the same time, the law clearly stipulates the legal responsibilities that offenders and institutions need to bear. A series of relevant national laws and regulations provide a legal basis for dealing with public emergencies in the Internet era. In the Internet age, from the perspective of content, the focus of public attention often becomes the stimulus for the emergence of public emergencies; the activities are characterized by online and offline group communication; online group activities have great influence and are difficult to manage.

The article "Analysis of News Dissemination Path and Impact of Big Data Technology in Public Health Emergencies" was retracted in 2023. Reasons: signs of a paper mill; suspected computer-generated content; unreliable results or conclusions; concerns about the data.

### 2.2. Emergency Preparedness for Public Health Events

#### 2.2.1. Emergency Prevention

(1) Awareness of emergency prevention: colleges and universities should pay special attention to emergency prevention, and establish a college emergency management team headed by the party secretary and chairman. Rescue operations should be carried out in a controlled manner, as quickly and efficiently as possible, to minimize accidents and minimize impact on victims and the emergency. (2) Strengthen control and management: on the other hand, it is necessary to further strengthen supervision and assessment, give full play to the role of the Disciplinary Committee in the inspection and control mechanism, and finally incorporate the special work of employees in emergencies into the employee assessment system. On the other hand, it is necessary to relieve pressure, share responsibilities, clarify task boundaries, establish and improve the accountability system, and express sincere congratulations to those who dare to take responsibility, dare to take responsibility, and dare to take responsibility in emergency situations to fulfill their obligations. For the relevant management departments or individuals who do not assume responsibility or do not act, they should conduct systematic screening and assign responsibility based on the best.

#### 2.2.2. Emergency Preparedness

(1) Strengthen emergency preparedness: establish and improve the guarantee reserve system for life-saving materials, training materials, training tools and equipment, and disposal facilities and equipment, improve the reserve system, and do a good job in the distribution of necessary medical equipment. The emergency facilities shall strengthen the management and control of the camp, ensure the complete supply of materials and equipment at reasonable prices, and ensure the timely delivery of valuables and valuables. (2) The safety of the program needs to be improved. When developing a rescue plan, the actual situation of the school should be considered, and coordination, safety, and accessibility should be fully considered. On the other hand, experts and researchers in the fields of safety management, emergency management, safety education and other fields inside and outside the school should be invited to conduct feasibility studies on the proposed scheme. On the other hand, it is necessary to further calibrate the effectiveness of rescue courses, carry out rescue plan drills in a timely manner, constantly find problems, correct the wrong, inaccurate and inappropriate parts of the rescue plan.

#### 2.2.3. Emergency Response

(1) Improve the emergency response mechanism: adhering to the principle of “people-oriented, prevention first” will greatly strengthen the establishment of social emergency measures, and truly develop an emergency response system, including “collaboration of the school, extensive participation of teachers and students, and strict prohibition on campus.” Work objective management. The second is the continuation of the “two shifts” in emergency management, that is, the whole process of management from one service to prevention, from disaster prevention and relief to postdisaster recovery. E-mail-based disaster response *H* mechanism from management to comprehensive management revises the emergency management system, and gradually establishes and improves a long-term emergency management mechanism. The third is to actively communicate with relevant ministries and commissions. Higher initiatives are based on the provincial emergency management system It is up to the government to establish a streamlined, systematic, and effective emergency management system in colleges and universities. (2) Improve the information exchange mechanism: the availability of information is a key factor in emergency situations. On the other hand, there is a need to create a single information platform through a coordinated emergency information system to effectively support information acquisition by universities and colleges. Feedback and monitoring procedures. On the other hand, technical tools such as information technology, artificial intelligence, and data analysis need to be strengthened to analyze, evaluate, and continuously monitor different situations. Identify areas of emergency and risk that may lead to social events and conduct accurate and timely analysis. As well as in the short-term emergency situation, the event carries on the monitoring, the forecast and the early warning forms the emergency processing mechanism. It is shown in Figure 1.

The article "Analysis of News Dissemination Path and Impact of Big Data Technology in Public Health Emergencies" was retracted in 2023. Reasons: signs of a paper mill; suspected computer-generated content; unreliable results or conclusions; concerns about the data.

### 2.3. Countermeasures for the Government to Properly Handle Public Emergencies

The Internet plays an important role in monitoring public opinion and provides a platform for ministries and commissions to effectively respond to emergencies. When dealing with emergencies, the government is in charge. In the Internet era, the government should properly handle public emergencies and focus on the following aspects.

#### 2.3.1. Mastering the Rules of News Release and Grasping the Initiative of the Right to Speak in the Process of Disposal

In the process of disposal, government departments should promptly announce the progress and truth of the incident. Public emergencies can easily arouse the public's strong demand for information. Only by truthfully releasing the progress of the incident to the public and satisfying the public's right to know to the greatest extent can the government firmly grasp the initiative of public opinion and occupy the mainstream public opinion field. At the same time, when government departments release information, they should try their best to use plain language and introduce them from the public's perspective. The practice of being arrogant and official will only arouse public disgust.

#### 2.3.2. Making Friends with the Media, Treating the Media Well, and Correctly Using and Guiding Public Opinion

Government departments should focus on mastering timeliness when dealing with the media. In an incident, the more scientific, professional, and transparent the government department handles the case, the more the mainstream media can get in touch with the case, and the ministries and the media can properly handle the case, deal with negative impacts, and actively communicate. Government departments should do a good job in information disclosure, improve information systems, and ensure smooth communication channels with the media; after public emergencies occur, government departments should promptly and proactively disclose to the media and society the dispositions at all stages, provided that they do not violate regulations situation, actively respond to media concerns, and consciously accept the supervision of public opinion.

The article "Analysis of News Dissemination Path and Impact of Big Data Technology in Public Health Emergencies" was retracted in 2023. Reasons: signs of a paper mill; suspected computer-generated content; unreliable results or conclusions; concerns about the data.

#### 2.3.3. Being Familiar with the Laws of Online Public Opinion and Cracking Down on Cyber Crimes in accordance with the Law

Practice has proven that open and transparent information is the best way to combat the root causes of the Internet. Therefore, government agencies need to establish mechanisms for timely information release and disclosure, relevant information release, online gossip monitoring, content verification, filtering, and technical means to deal with them to reduce negative public opinion.

#### 2.3.4. Enhancing the Sense of Responsibility of All Parties in Public Emergencies

The first is to establish a sense of responsibility of the government, the media, and the public “Trinity.” The government should clarify the identity of its own responsible subject and assume the main responsibility; the media should also shoulder the responsibility of disseminating information in the event; the public should understand their responsibilities in public emergencies, and do not believe or spread rumors. The second is to improve the accountability system. According to the responsibilities of each subject in the incident, legal procedures are initiated for irresponsible behaviors, it also strengthens accountability for relevant responsible persons and plays a warning role

## 3. Big Data Algorithms

### 3.1. Decision Unit Input and Output

We refer to inputs as “resources” consumed by political entities, such as inputs to factors of production. Instead, the output is the output of the decision unit, which represents the “efficiency level” after consuming a particular “resource.” Quantity, quality, and economic benefits of products. In general, when assessing the relative validity of data decay analyses, input and output variables should be out of bounds, free to omit, negative inputs, and positive outcomes. These two variables are initially independent variables, but in the binary data block analysis system, the same variable can be input or output, but belong to different stages and different decision-making units. Results and outputs are collectively referred to as the dimensions of the data model. Suppose there are *n* decision units in the evaluation system, each of which consumes *m* distinct inputs and produces *s* distinct outputs. Each decision unit is considered as a reference point, and the reference set is the collection of all reference points.

(1) $$\begin{array}{c} T=\left\{\left(x_{j},y_{j}\right)|j=1,\ldots ,n\right\},\\ T=\left\{\left(x,y\right)|x\in x_{j},j\in \left(1,\ldots ,n\right)\right\}. \end{array}$$

According to the axiom of triviality, different reference sets derived from different axiomatic assumptions are subsets of the possible output set. Satisfying all the above axioms is expressed as a continuous benchmark set:

(2) $$\begin{array}{c} T_{\text{crs}}=\left\{\left(x,y\right)|\sum_{j=1}^{n}\lambda_{j}X_{j}\leq X,\sum_{j=1}^{n}\lambda_{j}Y_{j},\;\lambda_{j}\geq 0\right\}. \end{array}$$

Another general assumption of the axiom is that the scaled return is a variable that satisfies the axioms of convexity, invalidity, triviality, and minima, and the corresponding reference data is represented as follows:

(3) $$\begin{array}{c} T_{\text{VRS}}=\left\{\left(x,y\right)|\sum_{j=1}^{n}\lambda_{j}X_{j}\leq X,\sum_{j=1}^{n}\lambda_{j}Y_{j}\geq Y,\sum_{j=1}^{n}\lambda_{j}=1\right\},\\ E_{0}=\text{Min}\theta_{o},\\ E_{0}=\text{Max}\sum_{r=1}^{s}u_{r}y_{r0}+u_{o}. \end{array}$$

Both of the above models are result-oriented BCC models, they keep the output constant and reduce the input as much as possible. When evaluating DEA performance, a DEA model is computed for each test unit and the DMUs that achieve different scores are ranked. Powerful units can also be divided into powerful and mild units, and the efficiency of each unit is calculated using the DEA model.

(4) $$\begin{array}{c} E\left(p,E\right)=\text{Min}\theta ,\\ E\left(\text{k,s}\right)=\min\theta_{k},\\ \phi \left(r,k\right)=\text{arcos}\left(\frac{\left(-x_{k},o\right),\left(x_{r}-x_{k}\right)}{\left(-x_{k},o\right)\times \left\|\left(x_{r}-x_{k}\right)\right\|}\right). \end{array}$$

The article "Analysis of News Dissemination Path and Impact of Big Data Technology in Public Health Emergencies" was retracted in 2023. Reasons: signs of a paper mill; suspected computer-generated content; unreliable results or conclusions; concerns about the data.

### 3.2. Optimization Check

After choosing the initial sample *S* and solving the model, it is also necessary to check whether the obtained efficiency is the value of the global efficiency, that is, whether the sample S already contains all the control points of the erroneous unit.

(5) $$\begin{array}{c} u^{*}y_{r}-v^{*}x_{r}\leq 0,\;\forall r\in s,\\ \lambda_{t}^{*}\left(u^{*}y_{r}-v^{*}x_{r}\right)=0,\;\forall r\in s. \end{array}$$

If, after solving the model, the selected sample finds that two of its dual factors do not satisfy the constraints, then we have not chosen its reference point for sample *S*, and the algorithm must redefine sample *S*. Therefore, we have to choose a new decision unit that is fairly comprehensive and will serve as a reference point for evaluating units, and insert S into the sample, removing the specific decision unit from the original sample to preserve sample size.

(6) $$\begin{array}{c} \begin{array}{cc} \text{s.t.} & AX=b,\;x\geq 0 \end{array}. \end{array}$$

The constraints are divided into two parts:

(7) $$\begin{array}{c} \text{Min}C^{T}X\\ \text{s.t.}A_{1}X_{1}=b_{1}. \end{array}$$

If the feasible region of the LP problem is bounded, we can represent *S* as a set of poles of a convex polygon. In the limiting case, we can convert LP to LP due to the convex joint principle.

(8) $$\begin{array}{c} \text{Min}\sum_{j\in J}C^{T}X^{j}\lambda_{j}. \end{array}$$

Use a column-generating algorithm to solve problems where there are far more such variables than the number of constraints. Usually there are many nodes in wholesale linear scale programming problems, and due to the large number of node elements in the convex complex set S, it is difficult for us to get these elements completely.

(9) $$\begin{array}{c} \text{Min}\sum_{k=1}^{p}\theta_{1}^{k}\lambda_{j}x_{ij}\leq \theta_{i}^{1}x_{io}\\ \sum_{j=1}^{n}\lambda_{j}=1,\;\lambda_{j}\geq 0,\;j=1,\ldots ,n. \end{array}$$

Based on this lemma, we solve LP, and the optimal solution obtained is also the original optimal LP solution. Therefore, we transform the original shell model into a diagonal structure LP and solve it with the DW decomposition algorithm.

(10) $$\begin{array}{c} \sum_{j=6}^{10}\lambda_{j}x_{ij}\leq \theta_{i}^{2}x_{i},\;\sum_{j=6}^{10}\lambda_{j}y_{rj}\geq y_{r}^{2},\;i=1,2,\;r=1,2,\\ \sum_{k=1}^{p}y_{ro}^{k}=y_{ro},\;r=1,\ldots ,s. \end{array}$$

This is basically the same as the DW decomposition algorithm, the only difference is how our algorithm is performed. We can get multiple poles of a subproblem to run the whole DW algorithm, but we use the Big-M method (penalty factor method) to execute the whole algorithm. In fact, in models to which DW decomposition algorithms can be applied, we usually take a few poles from each subproblem using heuristics or simple observations, and we use these poles to create the main program and its obstacles and solve them.

(11) $$\begin{array}{c} \left[\begin{array}{c} A_{1}\\ A_{2} \end{array}\right]=\left[\begin{array}{c} D_{1}D_{2}\\ F_{1}O\\ 0F_{1} \end{array}\right],\\ \begin{array}{cc} \text{Min} & \left(C^{T}-\pi A_{1}\right)X^{J}-a_{i}=\left[\begin{array}{c} A_{1}\\ A_{2} \end{array}\right] \end{array}. \end{array}$$

The article "Analysis of News Dissemination Path and Impact of Big Data Technology in Public Health Emergencies" was retracted in 2023. Reasons: signs of a paper mill; suspected computer-generated content; unreliable results or conclusions; concerns about the data.

## 4. News Dissemination Paths and Impact Analysis of Big Data Technology in Public Health Emergencies

### 4.1. Public Health Events under Big Data

Looking at the early warning work of previous public health crises, we can find shortcomings in early warning. At this stage of the early warning work, it is necessary to take targeted measures in the light of the specific circumstances of public health emergencies to improve the early warning mechanism for public health emergencies in our country and to improve work efficiency and hygiene accuracy. Early warning of emergencies can better protect citizens rights and interests and strengthen public order through early warning and the public interest. It is shown in Table 1.

From the data in Figure 2, FT-BERT-FC has the best average performance at 10-fold cross-validation. The macro-average *P*, macro-average *R*, and macro-average *K* are 0.619, 0.561, and 0.589, respectively. The second best performer is FT-GPT-FC with 0.598, 0.549, and 0.572 for *P*-mean macro, *R*-mean macro, and *K*!-mean macro, respectively. The better performance of FT-BERT-FC is due to the fact that BERT models with left-to-right and right-to-left transform structures are more efficient than GPT models with left-to-right transform structures.

From the data in Figure 3, we can see that the performance tests are different under different models. Under the big data model, the timeliness is 73.81%, the prudence is 84.25%, and the sustainability is 96.28%. Under the data mining model, the timeliness is 61.98%, the prudence is 77.58%, and the sustainability is 83.24%. The timeliness of the intelligent computing model is 53.44%, the prudence is 65.58%, and the sustainability is 96.28%. It can be seen that the timeliness, prudence, and sustainability of the big data model are compared with other models and performance has improved.

As we can see in the data in Figure 4, the total number of public health events has been increasing from 2015 to 2021. In 2015, there were 132 public sound events, with an increase of 8.9%; in 2016, there were 191 public sound events, with an increase of 12.3%; in 2017, there were 284 public sound events, with an increase of 15.79%; 368 cases with a growth rate of 17.21%; 473 cases of public sound events in 2019 with a growth rate of 19.87%; 501 cases of public health incidents in 2020 with a growth rate of 22.63%; and 573 cases of public health incidents in 2021 is 25.98%.

### 4.2. Analysis of News Dissemination Paths and Impacts in Public Health Emergencies

Public health emergencies are sudden major infectious diseases, large and unexplained diseases, serious food poisoning and occupational poisoning, etc., which have a serious impact on public health and may cause serious harm to public health. The new crown pneumonia epidemic first occurred in Wuhan City, Hubei Province, our country in late January 2020, and quickly spread to the whole country, and then to many countries around the world. It is a public health emergency. Public health emergencies are classified into four levels according to the nature, severity and extent of the emergency.

The article "Analysis of News Dissemination Path and Impact of Big Data Technology in Public Health Emergencies" was retracted in 2023. Reasons: signs of a paper mill; suspected computer-generated content; unreliable results or conclusions; concerns about the data.

From the data in Figure 5, we can see that in public health emergencies, the number of news dissemination paths including radio and television communication is 54 people, accounting for 13%; the number of digital TV broadcasters is 73 people, accounting for 19%; the number of public relations companies is 63 people, accounting for 16%; the number of people who reprint is 52 people, accounting for 12%; the number of people who search for communication is 73 people, accounting for 16%. It is 19%; the number of people who spread mobile phone text messages is 32, accounting for 9%.

The reliability coefficient of the data in Figure 6 is 0.950, which is greater than 0.9, indicating that the above survey data has high reliability for CITC analysis. A CITC score of 4 indicates a good level of confidence. Therefore, all the safety factors of the above study data are greater than 0.9, and the combination of different index values indicates that the data is highly reliable and can be used for further analysis. It is shown in Table 2.

As we can see in the data in Figure 7, the skill test was significant (chi = 425.364, *p* ≤ 0.001 < 0.05), which means that the selection ratio varied widely for each subject, and performance is compared based on differences in resonance or wear and differences in penetration levels. In particular, the response rate and prevalence were significantly higher for the 4 items of responsiveness, calmness, optimism, and hypervigilance.

## 5. Conclusion

By reviewing the previous work on early warning of public health emergencies, it is still possible to find gaps in early warning. Therefore, this paper takes the improvement of the early warning mechanism for public health emergencies as the breakthrough point, and combines the development and advancement of the early warning mechanism for public health emergencies in our country and the relevant legal framework to conduct a more detailed investigation of the current problems. This is a step forward in early warning and public health emergencies. According to the characteristics of public health events, we should improve the early warning mechanism of public health crisis in our country in a targeted manner, and improve the efficiency and accuracy of public health events. Public health emergencies are notified, and public order is consolidated through early warning to better protect public interests and individual rights.

The article "Analysis of News Dissemination Path and Impact of Big Data Technology in Public Health Emergencies" was retracted in 2023. Reasons: signs of a paper mill; suspected computer-generated content; unreliable results or conclusions; concerns about the data.

## Figures and Tables

**Figure 1:** Emergency preparedness for public health events.

**Figure 2:** Validation performance of public health events under different models.

**Figure 3:** Performance testing of public health events under different models.

**Figure 4:** The total number of public health events and their growth rates from 2015 to 2021.

**Figure 5:** News propagation paths and their proportions in public health events.

**Figure 6:** Analysis of the trust degree of news dissemination paths in public health events.

**Figure 7:** Summary graph of the influence rate and penetration rate of news dissemination.

**Table 1:** Validation performance of public health events under different models.

Methods	Macro-*P* average	Macro-*R* average	Macro-F1 average
Plain SVM	0.446	0.357	0.397
BOW-BIGRU-Att	0.54	0.439	0.484
WORD2VEC-BIGRU-Att	0.502	0.511	0.507
FastText-BIGRU-Att	0.542	0.52	0.531
GloVe--BIGRU-Att	0.56	0.517	0.538
ELMO--BIGRU-Att	0.577	0.537	0.561
FT-GPT-FC	0.598	0.549	0.572
FI-BERT-FC	0.619	0.561	0.589

**Table 2:** Analysis of the trust degree of news dissemination paths in public health events.

	CITC value	*a* coefficient	Cronbach coefficient
Highlight the emotional content of the event	0.673	0.947	0.897
Highlight the emotional content of the location	0.766	0.583	0.573
Highlight news and event topics	0.707	0.699	0.761
Highlight interpersonal emotional content	0.742	0.823	0.629
Highlight the emotional content of symbols	0.811	0.921	0.829
Highlight emotional choices for controversial events	0.761	0.747	0.921

## Data Availability

The experimental data used to support the findings of this study are available from the corresponding author upon request.
